# Antimycotic Activity of Some Medicinal Plants against *Mucor circinelloides*

**DOI:** 10.1155/2022/3523920

**Published:** 2022-02-25

**Authors:** Renu Jangid, Tahira Begum

**Affiliations:** Department of Botany, Samrat Prithviraj Chauhan Government College Ajmer, Rajasthan, India

## Abstract

The in vitro antimycotic activity of the leaf extract of *Catharanthus roseus*, *Lantana camara*, *Nerium indicum*, *Sida cordifolia*, and *Ziziphus mauritiana* was studied against *M. circinelloides*. This fungal species causes mucormycosis (black fungus). Presently, mucormycosis is affecting COVID patients due to prolonged use of steroids. So, it is needed to require development of more effective and less toxic antimycotic agents for the treatment of mucormycosis. Plants and their extraction preparations have been used as medicine against infectious disease. In this research, aqueous, ethanol, and DMSO (dimethyl sulfoxide) leaf extracts were used for antimycotic activity. All leaf extracts of selected medicinal plants recorded significant activity against *M. circinelloides*. Ethanol leaf extract of *C. roseus* showed the highest antimycotic activity followed by *N. indicum* and *L. camara. Z*. *mauritiana* which showed moderate activity against *M. circinelloides.*

## 1. Introduction

Plant products are an ample source of antimycotic drugs and are traditionally used for the treatment of various infectious diseases. A vast array of diseases occurs due to the fungal infections such as dermatophytosis, candidiasis, aspergillosis, and mucormycosis. Mucormycosis is an infectious disease caused by a fungus of the class of Zygomycetes and the order of Mucorales. *Mucor circinelloides* is one of the members of Zygomycetes that can cause mucormycosis (black fungus) in animals and humans. This fungus is ubiquitous and found in the environment and even in the nose and mucus of healthy people. It is thermotolerant and able to grow on a wide range of organic substrates and sporulates rapidly [1, 2].

In recent decades, the incidence of mucormycosis has increased all over the world, becoming the second most common fungal disease in patients with haematological malignancies and transplant recipients [3, 4, 5]. It affects the sinuses, the brain, and the lungs and can be life-threatening in diabetic or severely immunocompromised individuals. The different types of mucormycosis are classified according to the anatomic site of infection, such as rhino-orbital-cerebral, pulmonary, cutaneous, gastrointestinal, and disseminated infections [6].

Currently, doctors believe that mucormycosis is triggered by the use of steroids, a life-saving treatment for severely critically ill COVID-19 patients. Steroids reduce inflammation in the lungs for COVID. But they also reduce immunity and push up blood sugar levels in both diabetics and nondiabetic COVID-19 patients. It is thought that this drop in immunity could be triggering cases of mucormycosis.

Recently, the use of some natural plant products has emerged to inhibit the causative organisms. Plant products are major sources of therapeutic drugs for infectious disease and commonly harmless or have the least side effects as compared to synthetic drugs [7, 8]. Testing leaf extracts of medicinal plants for antimycotic activity could be a good source to identify new antimicrobial drugs.

The aim of this study was to assess the antimycotic activity of leaf extracts of five medicinal plants including *Catharanthus roseus*, *Lantana camara*, *Nerium indicum*, *Sida cordifolia*, and *Ziziphus mauritiana* against *Mucor circinelloides*.

## 2. Material and Methods

### 2.1. Fungal Material

*Mucor circinelloides* culture was isolated from soil samples by hair baiting technique [9]. The culture was authenticated by the Indian Agriculture Research Institute (IARI), Delhi. The isolated fungus culture was maintained on Sabouraud's Dextrose Agar (SDA) medium (Figures 1 and 2).

### 2.2. Plant Material

The present investigation deals with the screening of leaf extracts of selected five medicinal plants *Catharanthus roseus*, *Lantana camara*, *Nerium indicum*, *Sida cordifolia*, and *Ziziphus mauritiana* for antimycotic activity. Leaves were collected from the local area of Ajmer district, Rajasthan, and authenticated by the Department of Botany, Samrat Prithviraj Chauhan Government College Ajmer, Rajasthan, India. The leaves were washed thoroughly 2-3 times with running tap water and dried in the shaded area. After then, dried plant material was ground into powder using a blender and sealed in polythene bags for further use.

### 2.3. Preparation of Leaf Extracts

Leaf extract was prepared by Soxhlet extraction method [10]. About 20 g of dried powdered leaf material was uniformly packed into a thimble and run in Soxhlet extractor with ethanol or DMSO (dimethyl sulfoxide) for 48 hours. The extract was then filtered with the help of filter paper, and solvent was evaporated from the extract. For aqueous extraction, 20 g of powdered plant material was macerated by a blender with 200 ml of distilled water and the solvent powder mixture was kept at room temperature for 48 hours; the extract was filtered through filter paper. The extracts were kept in the refrigerator at 40°C for further experiments.

### 2.4. Preliminary Phytochemical Screening

The preliminary phytochemical testing of leaf extracts to detect the presence of different secondary metabolites was done. Air-dried and powdered leaf materials were screened for the presence of alkaloids, flavonoids, phenols, terpenoids and steroids, proteins, amino acids, saponin, reducing sugar, and glycoside compounds as described in literature. The ethanolic leaf extracts of selected medicinal plants were tested for preliminary phytochemical screening using basic standard procedures [11].

### 2.5. Antimycotic Activity

The antimycotic study of leaf extracts of selected medicinal plants was determined by using the disc diffusion method [12]. Filter paper discs of 6 mm diameter were soaked with 1 ml of extracts. Sabouraud's Dextrose Agar (SDA) plates were inoculated with *M. circinelloides* culture by point inoculation. The plates were done in triplicates and were incubated at 28°C. The antimycotic activity was taken on the basis of diameter of zone of inhibition, which was measured after 7 days of incubation, and the mean of three readings is presented.

### 2.6. Control Experiment

The presence of the inhibition zone of the selected fungus was calculated using griseofulvin as standard.

### 2.7. Statistical Analysis

The data were analysed using one-way analysis of variance (ANOVA) and calculated as mean ± SD.

## 3. Results

### 3.1. Preliminary Detection of Phytocompounds

The data on phytochemical analysis showed both presence and absence of various compounds (Table 1). The preliminary detection of phytochemical present in leaf extracts of *Catharanthus roseus*, *Lantana camara*, *Nerium indicum*, *Ziziphus mauritiana*, and *Sida cordifolia* showed positive results for most of the phytochemical constituents, namely, alkaloids, flavonoids, phenols, terpenoids and steroids, proteins and amino acids, saponin, reducing sugar, and glycosides.

### 3.2. Antimycotic Activity of Selected Medicinal Plants

The antimycotic activity of different leaf extracts against *M. circinelloides* was evaluated by the disc diffusion method. The results and screening of antimycotic activity of leaf extracts of *Catharanthus roseus*, *Lantana camara*, *Nerium indicum*, *Sida cordifolia*, and *Ziziphus mauritiana* are summarized in Table 2. All the extracts tested exhibited different degrees of antimycotic activity against *M. circinelloides*. The ethanol leaf extract of *C. roseus* and *N. indicum* showed the highest antimycotic activity with zone of inhibition 23 mm and 22 mm, respectively. *S. cordifolia* and *Z. mauritiana* showed moderate activity against *M. circinelloides*. The aqueous leaf extract of *N. indicum* and *C. roseus* showed maximum activity (20 mm, 19 mm) against *M. circinelloides*. DMSO extracts of all selected plants showed good antimycotic activity except *Z. mauritiana*. The percentage of growth inhibition of the selected medicinal plants was recorded, and the data are shown in Table 3. The percentage growth inhibition of pathogenic fungi by leaf extracts was data put in a graph present in Figure 3. The graph showed that ethanol leaf extract exhibited strong antimycotic activity. The highest percentage zone of inhibition was shown by ethanol leaf extract of *C. roseus* (96%) and moderate by aqueous extract of *S. cordifolia* (58%) and DMSO extract of *Z. mauritiana* (58%).

Inhibition zone of griseofulvin = 24 mm.

## 4. Discussion

Recently, a number of mucormycosis (black fungus) cases are being detected among COVID-19 patients in some states of India including Delhi, Maharashtra, and Gujarat. According to Dr. Mahesh (Consultant, Department of Internal Medicine, Narayana Health City, Bengaluru), mucormycosis can be very dangerous; if left untreated, it can cause mutilating damage to the face, nose, and eyes with disfigurement and loss of vision and also cause invasive brain infection (Dr. Mahesh).

A review of literature indicates that the plant has been studied with respect to its antimicrobial properties. Phytochemicals including alkaloids, flavonoids, phenols, terpenoids and steroids, proteins and amino acids, saponin, reducing sugar, and glycosides were known to possess antimycotic activity. Therefore, this study focuses on the antimycotic properties of leaf extracts. *C. roseus* showed the presence of many alkaloids, and they are responsible for many medically important activities of this plant such as antibacterial, anticancer, antifungal, antidiabetic, and antiviral activities [13]. The methanol leaf and flower extracts of *Lantana camara* showed antifungal activity (20 mm) against dermatophytes [14]. The ethanol extract of *N. indicum* leaves showed antifungal activity against *Aspergillus niger* and *Candida albicans* with zone of inhibition of 10 mm and 13 mm, respectively [15]. The phytochemical screening and *in vitro* efficacy of antimicrobial activities of chloroform leaf extract of *Sida cordifolia L.* were studied against some human pathogenic bacterial and fungal strains [16]. The extracts of some *Cassia*, *Detarium*, and *Ziziphus* species showed antifungal activity against dermatophytes [17].

In the present work, ethanol leaf extract of *C. roseus* was shown to have maximum activity against *M. circinelloides*. The leaf extract of *Z. mauritiana* showed the least activity against *M. circinelloides*. The result of the present investigation clearly indicates that the antimycotic activity varies with the species of plants and plant products used. Thus, they ascertain the plants used in Ayurveda, which could be of considerable interest to the development of new drugs.

## 5. Conclusion

The conclusion of this study supports the traditional medicinal use of various plant extracts (*Catharanthus roseus*, *Lantana camara*, *Nerium indicum*, *Sida cordifolia*, and *Ziziphus mauritiana*) in treating infectious diseases, at present, of those people suffering from mucormycosis who had recovered from COVID-19. An overall mortality rate of 50% may be being triggered by the use of steroids, a life-saving treatment for critically ill COVID-19 patients. Therefore, this study focuses on the antimycotic properties of leaf extracts which are used to develop natural drugs.

## Figures and Tables

**Figure 1:** *M. circinelloides* culture.

**Figure 2:** Microscopic structure.

**Figure 3:** In vitro antifungal activity of leaf extracts of some medicinal plants against *M. circinelloides*.

**Table 1:** Preliminary phytochemical screening of ethanolic leaf extracts of selected medicinal plants.

S. no.	Test	*Catharanthus roseus*	*Lantana camara*	*Nerium indicum*	*Sida cordifolia*	*Ziziphus mauritiana*
1	Alkaloids	+	+	+	+	−
2	Flavonoids	+	+	+	+	+
3	Phenolic compounds	+	+	+	+	+
4	Terpenoids and steroids	+	+	+	+	+
5	Proteins and amino acids	+	+	+	+	+
6	Saponins	+	+	+	+	+
7	Reducing sugars	+	+	+	+	+
8	Glycosides	+	+	+	+	+

**Table 2:** Antimycotic activity of leaf extracts of some medicinal plants against *Mucor circinelloides*.

S. no.	Plants	Zone of inhibition		
		Aqueous	Ethanol	DMSO
1	*Catharanthus roseus*	19 ± 1.1	23 ± 0.5	20 ± 0.5
2	*Lantana camara*	18 ± 0.5	21 ± 0.5	18 ± 1.1
3	*Nerium indicum*	20 ± 0.5	22 ± 0.5	20 ± 1.1
4	*Sida cordifolia*	14 ± 1.1	16 ± 1.1	19 ± 0.5
5.	*Ziziphus mauritiana*	16 ± 1.1	15 ± 0.5	14 ± 0.5

**Table 3:** The % inhibition of the different plant extracts compared to griseofulvin (100% inhibition) against *M. circinelloides*.

S. no.	Plants	% growth inhibition			
		Griseofulvin	Aqueous	Ethanol	DMSO
1	*Catharanthus roseus*	100	79	96	83
2	*Lantana camara*	100	75	88	75
3	*Nerium indicum*	100	83	92	83
4	*Sida cordifolia*	100	58	67	79
5	*Ziziphus mauritiana*	100	67	63	58

## Data Availability

Data are attached in the manuscript.

## References

[1] Richardson M. (2009). The ecology of the Zygomycetes and its impact on environmental exposure. *Clinical Microbiology and Infection*.

[2] Ingold C. T. (1978). The Biology of Mucor and Its Allies. *Studies in biology no. 88*.

[3] Kontoyiannis D. P., Lionakis M. S., Lewis R. E. (2005). Zygomycosis in a tertiary-care cancer center in the era of Aspergillus-active antifungal therapy, a case-control observational study of 27 recent cases. *The Journal of Infectious Diseases*.

[4] Lanternier F., Sun H. Y., Ribaud P., Singh N., Kontoyiannis D. P., Lortholary O. (2012). Mucormycosis in organ and stem cell transplant recipients. *Clinical Infectious Diseases*.

[5] Lewis R. E., Kontoyiannis D. P. (2013). Epidemiology and treatment of mucormycosis. *Future Microbiology*.

[6] Spellberg B., Edwards J., Ibrahim A. (2005). Novel perspectives on mucormycosis: pathophysiology, presentation, and management. *Clinical Microbiology Reviews*.

[7] Clardy J., Walsh C. (2004). Lessons from natural molecules. *Nature*.

[8] Bhadauria S., Kumar P. (2011). In vitro antimycotic activity of some medicinal plants against human pathogenic dermatophytes. *Indian journal of fundamental and Applied Life Sciences*.

[9] Harborone J. B. (1973). *Phytochemical Methods Chapman and Chapman*.

[10] López-Bascón M. A., Luque de Castro M. D. (2020). *Liquid phase extraction*.

[11] Harborne J. B. (1998). *Phytochemical Methods-A Guide to Modern Techniques of Plant Analysis*.

[12] Kirby W. W. M., Yoshihara G. M., Sundsted K. S., Warren J. H. (1956). *Clinical usefulness of a single disc method for antibiotic sensitivity testing*.

[13] Patil P. J., Ghosh J. S. (2010). Antimicrobial activity of Catharanthus roseus – a detailed study. *British Journal of Pharmacology and Toxicology*.

[14] Bokhari F. M. (2009). Antifungal activity of some medicinal plants used in Jeddah, Saudi Arabia. *Mycopathologia*.

[15] Kalita D., Saikia J. (2012). Ethnomedicinal, antibacterial and antifungal potentiality of *Centella asiatica*, *Nerium indicum* and *Cuscuta reflexa*-widely used in Tiwa tribe of Morigaon district of Assam, India. *Int J Phytomedicine*.

[16] Venkatachalam D., Thavamani S., Sebastian A. C. (2019). Evaluation of antimicrobial activity of Sida cordifolia leaf extract. *South Asian popular culture*.

[17] Adamu H. M., Abayeh O. J., Ibok N. N., Kafu S. E. (2006). Antifungal activity of extracts of some Cassia, Detarium and Ziziphus species against dermatophtyes. *Natural product radiance*.

